# Optimal Medical Image Size Reduction Model Creation Using Recurrent Neural Network and GenPSOWVQ

**DOI:** 10.1155/2022/2354866

**Published:** 2022-02-26

**Authors:** Chethana Sridhar, Piyush Kumar Pareek, R. Kalidoss, Sajjad Shaukat Jamal, Prashant Kumar Shukla, Stephen Jeswinde Nuagah

**Affiliations:** ^1^Department of Computer Applications, Sivananda Sarma Memorial R.V. College, Bangalore, Karnataka, India; ^2^Department of Computer Science Engineering, Nitte Meenakshi Institute of Technology, Bangalore, Karnataka, India; ^3^Sri Sivasubramaniya Nadar College of Engineering, Chennai, India; ^4^Department of Mathematics, College of Science, King Khalid University, Abha, Saudi Arabia; ^5^Department of Computer Science and Engineering, Koneru Lakshmaiah Education Foundation, Vaddeswaram, Guntur 522502, Andhra Pradesh, India; ^6^Department of Electrical Engineering, Tamale Technical University, Tamale, Ghana

## Abstract

Medical diagnosis is always a time and a sensitive approach to proper medical treatment. Automation systems have been developed to improve these issues. In the process of automation, images are processed and sent to the remote brain for processing and decision making. It is noted that the image is written for compaction to reduce processing and computational costs. Images require large storage and transmission resources to perform their operations. A good strategy for pictures compression can help minimize these requirements. The question of compressing data on accuracy is always a challenge. Therefore, to optimize imaging, it is necessary to reduce inconsistencies in medical imaging. So this document introduces a new image compression scheme called the GenPSOWVQ method that uses a recurrent neural network with wavelet VQ. The codebook is built using a combination of fragments and genetic algorithms. The newly developed image compression model attains precise compression while maintaining image accuracy with lower computational costs when encoding clinical images. The proposed method was tested using real-time medical imaging using PSNR, MSE, SSIM, NMSE, SNR, and CR indicators. Experimental results show that the proposed GenPSOWVQ method yields higher PSNR SSIMM values for a given compression ratio than the existing methods. In addition, the proposed GenPSOWVQ method yields lower values of MSE, RMSE, and SNR for a given compression ratio than the existing methods.

## 1. Introduction

Modern learning reports that the employment of imaging has increased significantly in the previous two decades [1]. In the United States, for example, there was a study by Smith-Brinman et al. [2]. It was reported in 2008 that CCTV images doubled and MRI images doubled. This growth is the effect of a quick overhaul of hardware as well as software to support imaging systems. In addition, the transition from analog to digital provides fast, stress-free, and accurate image development. All of these factors have supplied significantly to the group of images. Therefore, the byte of these images is received every year worldwide. Imaging technology is implemented by X-ray, ultrasound, MRI/fMRI (functional magnetic resonance image), nuclear medicine, PET (positron emission tomography), CT (computerized tomography) [3], and DXA (dual energy X-ray absorptiometry). The necessity of saving, distributing, and downloading these images in their own appearance has given to the picture archiving along with communication system (PACS) a medical imaging skill that presents low-cost storage as well as access to useful images from many sources. Unluckily, the huge pixel size of these images severely limits the storage capacity [4–6]. For example, an emblematic NMR matrix dimension is 512 × 512 with 16 b [7].

A healthcare association that creates hundreds of images a week will need numerous megabytes of storage space. In a year, the total storage needed increases to a few gigabytes. This growth results in various terabit storage volumes per year. Moreover, a 56 kbps MRI band will take 12–15 minutes [8]. A lot of methods have been developed to reduce the size of these images, except that the major desirable novelty is the hybrid image production technique, in which the wavelet transform (DWT) along with vector quantization (VQ) as well as the loss [9] is preferred the most. In numerical analysis and function, DDD is a variation of spectacles in which the spectacles are precisely modeled and designed to process signals with a certain amount of time [10, 11].

In contrast to the discrete cosine transform (DCT) derived from the function of the base cosine, DWT is able to collect a few functions that meet the needs of multidimensional reaction analysis [12]. The origin of the image size reduction algorithm is to get an *X* input as well as produce an *X* demonstration that must need less bits for the representation. This went after recovery techniques that work on a compact X representation to produce a recovery , e.g., DWT offers a set of wavelet coefficients at various sizes showing various numerical types.

To propose the quantity for every set using the VQ technique, the bit value can significantly condense, devoid of affecting the excellence. Nevertheless, quantification leads to defeat of signal superiority. Consistent with Sannon, the dimensions of the selected vector have a significant influence on the quantitative efficiency. Larger vectors produce better quality than smaller vectors. For this reason, the purpose of this work is to develop a hybrid approach derived from discrete wavelet transforms and vector quantization to reduce the size of medical images with elevated compression rates and quality.

The main contributions of this paper are summarized as follows:

- Recurrent neural network is developed to compress the medical images.
- A novel hybridized approach GENPSO is developed for optimizing the neural network parameters.
- Using GENPSO, the hidden layer of recurrent neural network is compressed in more effective way to increase the compression ratio.
- High compression ratio and better performance were achieved compared to the other existing approaches using wavelet vector quantization.
- The proposed method provides good results for real-time medical dataset.

The manuscript of this document is organized as follows: Section 2 discusses some of the relevant contemporary literature.  Section 3 presents a detailed description of the proposed architecture.  Section 4 presents the experimental results, which include the general operating results of comparing the performance of GENPSO and other compression methods previously published. Conclusion and future work are provided in Section 5.

## 2. Background

Juliet et al. [13] discussed a new approach, including Ripplet conversion, to ensure better image quality and higher compression levels. In this work, to achieve high compression, the image is presented in various weights and instructions. Cyriac et al. [14] developed a lossless compression technique to address the issue of expanding compression. In this article, the newly developed method is to reduce the image size sufficiently as well as speed up the hardware execution of the software in real time. Brahimi et al. [15] illustrated a new coding method in which both symbols along with images are compressed together with a codec. The major point of this method is to insert a rotten stray signal into the corrupted image, and the resulting image is employed for image size reduction.

Arif et al. [16] introduced an effective approach for minimizing fluoroscopic imaging. The retrieved ROI of this approach is minimized through a grouping of run length as well as hepatic coding. The final outputs show that the newly developed method offers a compression ratio of 400% compared to other traditional approaches. Das et al. [17] described a lossless medical imaging watermark (MIW) procedure that relies on the area of interest concept. The major purpose of this technique is to offer clarification to many issues related to the dissemination of medical data. This article uses seven various methods to display as well as compare outputs to demonstrate that the newly developed approach is easy and obvious in ensuring the security of the medical database.

Lucas et al. [18] introduced 3D lossless compression techniques 3-D MRP for high-volume medical imaging equipment. The presented technique relies on the minimum velocity forecasting mechanism (MRP). This article concludes that the demonstrated method can enhance the probability of error of the MRP as well as achieve higher image size reduction efficiency than ASS along with other standards for the depth of the medical signal. Špelič et al. [19] proposed new algorithms developed as voxel compression algorithms for 3D CT image compression for the broadcasting of graphics information acquired from CT scanners. This work illustrated the Hounsfield size being employed first for partial medicine, and then image size reduction is applied. In this work, a modeling method is employed to evaluate the effectiveness of the newly developed techniques.

Anusuya et al. [20] developed a new, lossless code employing a codec to reduce the size of 3D brain images. In this paper, MRI models are employed to analyze the effectiveness of the newly developed solution, and this paper focuses on sinking utilization time using parallel calculations. Xio et al. [21] introduced integrated tablets for compact image compression without data loss. The proposed technique integrates with integer maps for inefficient compaction. Amri et al. [22] introduced two lossless image size reduction techniques. In this work, demonstrated algorithms are employed to minimize image dimension and code algorithms for lossless image size reduction. It can be seen that the newly developed method can maintain image feature for elevated image size reduction levels and also provide different enhancements to the standard JPEG image size reduction.

Ramesh et al. [23] described a method for predicting wavelengths to minimize medical images. In this method, the forecast equations for each subline depend on the correlation analysis. Evaluation outputs show that the newly developed method offers a superior level of compression matched up to the standard SPHIT and JPEG2000. Ibrahim et al. [24] introduced two novel lossless image size reduction techniques based on logarithmic calculations. The proposed method can offer better image feature compared to conventional DWT. Avramovic et al. [25] developed a new loss-free image size reduction technique using context-based Internet converters. The proposed method relies on the concept of projection to eliminate the need for transparency in the image and to effectively compress the image without losing data. The conclusion is that the newly developed method can attain the similar results as high-class images like previous standard algorithms. Bairagi [26] accounted the idea of symmetry for medical imaging. The method shown here is lossless and can effectively remove unnecessary information from the image.

Zuo et al. [27] introduced an enhanced technique to IMIC-ROI medical imaging for efficient and effective medical imaging. The proposed technique is based on the concept of interest area (ROI) as well as non-ROI area. Srinivasan et al. [28] described encoders for compact electromagnetism (EEG) matrix. The method illustrated first two phases, the lost code layer (SPHIT) and the remaining coded layer. Taquet et al. [29] reported on hierarchical-oriented forecasting methods to allow scaling without loss and near-loss of medical imaging. It can be seen that the newly developed method is best employed for lossless image size reduction as it may offer superior or equivalent PSNR for higher bit rates compared to the JPEG 2000 standard.

Zanaty and Ibrahim [30] introduced a medical image compression technique based on combining region growing and wavelets algorithms. The authors have used a region growing algorithm where an image is portioned into two parts and the capability of the algorithm is justified.

## 3. Materials and Methods

### 3.1. Recurrent Neural Network

The recurrent neural network [31] is one of the neural networks which employs precedent data in a closed loop. It can be repeated through merely transmitting the network output or intermediate state as input. For instance, the input image of k-1 might be integrated into a network in kth step. This kind of network is suitable during short-term dependencies as it depends on other and does not perform better for long-term dependencies observed in compression. For this kind of network, there are issues in the training procedure, so throughout reproduction it can “disappear” or “explode.” To avoid this limitation, this work uses a new approach called GenPSO and proposed vector quantization required to incorporate with neural network to manage the input and output image data. So in this work the codebook is generated using a novel hybrid GenPSO approach. Then this codebook is used in vector quantization for compressing the number of hidden neurons for increasing the compression ratio [32].

### 3.2. Updating Weights in Recurrent Neural Network Using GenPSO

In this step, the weight generated from the recurrent neural network is updated through the GenPSO method. The initial constitutive population of a chromosome has an evenly distributed random number. The chromosome represents the weight of the recurrent neural network. A crossover here can be defined as a crossover on a node. It is necessary to construct two springing from the parent node, with each node being retrieved from a hidden layer, and multiple outputs, randomly taken with equal probability. This node is considered a transit node [33]. The value of all input weights for that particular node is changed with the other master. This change can also be considered as a node change, in which all the incoming weights are for randomly selected active nodes. Finally, the PSO process is applied. The initial PSO population was determined by GA decision. Therefore, it can overcome the problem of slow convergence of the GPS network [34].

The algorithm for weights evolution by GenPSo in RNN is as follows.

The following steps are performed to determine the best weight value.

- For population of the XiMi, a solution, *i* = 1,…, *μ*, is started on area *M* with *R*∈*n*.
- Two parents are randomly selected with a parent population distribution and two births will be generated by a crossover operator.
- ereditary mutation of the offspring is performed.
- Repeat step (ii) until the number of offspring *μ*o is *μ*. Otherwise, go to step (v).
- Any parental decision, *i* = 1,…, *μ* and progeny Xo, *o* = 1,…, *μ*, are estimated in light of objective function (*X*).
- For mixed population Xm, m = 1,…, 2 *μ*, both the parent population and the population formed. They are randomly mixed so that parents and children mix up properly.
- Each solution of Xm, *m* = 1,…, 2 *μ* is evaluated with 10% of the solutions of the other randomly selected solutions from a mixed population.
- The highest earnings decision is reserved for the next generation of parents.
- If the best chromosome difference for the N number of successive generations is less than the specified brightness, stop the process and the best chromosome of the last generation is the ideal weight. Otherwise, proceed to the next step.
- Beginning particle population and location and velocity are derived from the genetic algorithm.
- Estimate the fitness value of all particles depending on the fitness function based on the objective of the optimization problem.
- Compare the values of the fit of each particle and its holes. If the current value is better than pbest, then set the current fitness value to its pbest. Otherwise, the pbest will remain the same.
- Determine the current best fitness value among all fitness values of all particles in the population. Then, compare this value to Gebel and set the current value to Gebel if the current value is better than Gebet. Otherwise, leave it blank.
- Update the position and speed of each piece.
- Stop if the best solution is found that matches the predefined minimum error or reaches the maximum number of repetitions. Otherwise, repeat the procedure from steps (x) to (xv).

### 3.3. Proposed Image Compression Using GenPSO Wavelet Vector Quantization Recurrent Neural Network Approach

The proposed technique for quantifying vectors using backward neural networks is summarized in the following steps:

**Step 1 .**

Apply wavelet transform to the image to produce transformed image.

**Step 2 .**

Get a pixel value (0 to 255) of the matrix.

**Step 3 .**

Now apply these values to the forward neural network. This network must have 64 input nodes since the detector is 8 × 8. Train the recurrent neural network using the training algorithm as explained in Section 3.2.

**Step 4 .**

Weight and tilt, updated by GPS, are fed to a hidden layer that can contain 2, 4, 8, 16, 32, and 64 hidden nodes. Encode these values with GenPSOWVQ

**Step 5 .**

Select the 8 × 8 printer in order after completing the training.

**Step 6 .**

Digital bits are now converted into real values.

**Step 7 .**

Finally, the call phase shows depressed images (output images) at the output of the nervous system's output layer. The conversion of a pixel to a true value and a true value to a pixel occurs during the compression and compression process.

## 4. Experimental Results

### 4.1. Dataset Used

Datasets of images which include chest radiographs, unenhanced brain CTs, mammograms, and abdominal CTs are used for experimenting this work. The performance of the proposed Int OPMICM method is evaluated using real-time medical images in terms of PSNR, MSE, SSIM, NMSE, SNR, and CR values [31]. These results are compared with those obtained by the existing algorithms, namely, FFNN, VQFFNN, optimized FFNN, and optimized VQFFNN.  Figure 1 depicts the sample images from the real-time medical database [34].

### 4.2. Performance Metric

For the assessment of the compression approaches, this paper employs six metrics, namely, PSNR, MSE, SSIM, NMSE, SNR, and CR.

#### 4.2.1. Peak Signal-to-Noise Ratio

The peak signal-to-noise ratio (PSNR) is used to evaluate the quality between the compressed image and the original image. The PSNR formula is defined as follows:

(1) $$\begin{array}{c} \log\;10\frac{255\times 255}{1/H\times W\sum_{x=0}^{H-1}\sum_{y=0}^{W-1}{\left[f\left(x,y\right)-g\left(x,y\right)\right]}^{2}}\text{d}B, \end{array}$$

where *H* and *W* are the height and width of the image, respectively, and *f*(*x*, *y*) and *g*(*x*, *y*) are the grey levels located at coordinate (*x*, *y*) of the original image and compressed image, respectively.

#### 4.2.2. Structural Similarity Index

The structural similarity index is a method for measuring the similarity between the compressed image and the original image.

(2) $$\begin{array}{c} SSIM\left(y,\;\hat{y}\right)=\;\frac{\left(2_{\mu_{y}\mu_{\hat{y}}}+\;c_{1}\right)\left(2\sigma_{y\hat{y}}+\;c_{2}\right)}{\left(\mu_{y}^{2}+\;\mu_{\hat{y}}^{2}+\;c_{1}\right)\left(\sigma_{y}^{2}+\;\sigma_{\hat{y}}^{2}+\;c_{2}\right)}, \end{array}$$

where $\hat{Y}$ is the compressed image, *Y* is the original image, *μ* is the mean, and *σ^2^* is the variance.

#### 4.2.3. Mean Square Error

The mean square error (MSE) is used to evaluate the difference between a compressed image and the original image. The MSE can be calculated by

(3) $$\begin{array}{c} \text{MSE}=\;\frac{1}{n}\overset{n}{\underset{i=1}{\sum }}{\left({\hat{Y}}_{i}-Y_{i}\right)}^{2}, \end{array}$$

where $\hat{Y}\hat{Y}$ is the compressed image and *Y* is the original image.

#### 4.2.4. Root Mean Square Error

The root mean square error (RMSE) is a frequently used measure of the difference between compressed image values and the original image values.

(4) $$\begin{array}{c} \text{RMSE}=\;\sqrt{\frac{\sum_{i=1}^{n}{\left({\hat{Y}}_{i}-Y_{\;i}\right)}^{2}}{n}}, \end{array}$$

where $\hat{Y}\hat{Y}$ is the compressed image and *Y* is the original image.

### 4.3. Experimental Analysis

#### 4.3.1. Experiment No. 1: Analysis of the Proposed GenPSOWVQ Compression Approach

In this experiment, we will evaluate the contribution of the proposed GenPSOWVQ compression approach. To evaluate the performance of this scheme, the PSNR, MSE, SSIM, NMSE, and SNR against 25% CR ratio are employed. This is shown in equations (1)–(4) correspondingly. This experiment will introduce the concept of GenPSOWVQ compression. It will be performed by estimating the performance of this scheme against a 25% CR ratio.  Table 1 lists the PSNR, MSE, SSIM, NMSE, and SNR measures of GenPSOWVQ as well as the existing approaches.

The proposed GenPSOWVQ approach's performance is compared with traditional compression approaches through varying metrics, and the result is illustrated in Figure 2. The performance ratio of GenPSOWVQ has higher value than with traditional compression approaches. So it is proved that GenPSOWVQ is superior to traditional compression approaches.

#### 4.3.2. Experiment No. 2: Performance of Best Chromosome Particles of GenPSO with Population Size of 50

The designed 2-2-1 feed forward architecture and the error value were developed according to the GenPSO method set out above. The population size was 50, and the termination rule is if the best error in the chromosome in the 50 successive generations is less than 0.00001. It is described in Figure 3.

The proposed GenPSO approach's performance is compared with varying population size, and the result is illustrated in Figure 3. The performance ratio of GenPSO has higher value than with traditional compression approaches. So it is proved that GenPSOWVQ is superior to traditional compression approaches.

#### 4.3.3. Experiment No. 3: Performance of Best Chromosome Particles of GenPSO with Population Size of 100

The architecture of the best chromosome particle [35] distribution 2–2–1 was developed using the GenPSO method described above. The population size was 100, and the termination rule is if the 100 best chromosome errors continue to be less than 0.00001. It is described in Figure 4.

The proposed GenPSO approach's performance is compared with varying population size of 100, and the result is illustrated in Figure 4. The performance ratio of GenPSO has higher value than with traditional compression approaches. So it is proved that GenPSOWVQ is superior to traditional compression approaches.

#### 4.3.4. Experiment No. 4: Performance of Error of GenPSO with Population Size of 50

The designed 2-2-1 feed forward architecture and the error value were developed according to the GenPSO method set out above. The population size was 50, and the termination rule is if the best error in the chromosome in the 50 successive generations is less than 0.00001. It is described in Figure 5.

The proposed GenPSO approach's performance is compared with varying population size of 50, and the result is illustrated in Figure 5. The performance ratio of GenPSO has higher value than with traditional compression approaches. So it is proved that GenPSOWVQ is superior to traditional compression approaches [36]. The proposed GenPSO achieves high performance against a large population size. This shows that it is superior to traditional compression approaches.

## 5. Conclusion

This article presents an image compression method for medical image compression using recurrent neural network. This recurrent neural network used a new image compression scheme called the GenPSOWVQ method which has been introduced using GenPSO with wavelet VQ. The codebook is built using a combination of fragments and genetic algorithms. The proposed method was tested using real-time medical imaging using PSNR, MSE, SSIM, RMSE, SNR, and CR indicators. Experimental results show that the proposed GenPSOWVQ method yields higher PSNR SSIMM values for a given compression ratio than the existing methods. In addition, the proposed GenPSOWVQ method yields lower values of MSE, RMSE, and SNR for a given compression ratio than the existing methods. This work can be further expanded to achieve the goal of creating optimal rules. The work can be extended for security in case of image compression. Like the future work for this work, a new code of image compression is proposed using ambiguous logic. This research work has to be tested on large datasets and on a dynamic huge sample that is not tested and storage optimization that is not considered. The article presents a method for image compression using a recurrent neural network known as GenPSO. This method is built using a combination of genetic algorithms and fragments. The test results indicated that the proposed method achieves higher PSNR SSIMM values than the existing methods.

## Figures and Tables

**Figure 1:** Experimental images.

**Figure 2:** Analysis of PSNR, MSE, SSIM, NMSE, and SNR of GenPSOWVQ approach along with 25% CR ratio.

**Figure 3:** Analysis performance of best chromosome particles.

**Figure 4:** Analysis performance of best chromosome particles with 100 iterations.

**Figure 5:** Analysis performance of best chromosome particles with population size of 50.

**Table 1:** Analysis of PSNR, MSE, SSIM, NMSE, and SNR of GenPSOWVQ approach along with 25% CR ratio.

Dataset					
Compression approaches					
Metrics	OFFNN	VQFFNN	VQOFFNN	IntOPMICM	GenPSOWVQ
PSNR	36.80	48.12	49.65	52.4227	60.64
SSIM	0.20	0.43	0.53	0.6736	0.86
MSE	13.57	8.86	6.19	1.4164	0.83
RMSE	3.68	0.001	2.48	1.1901	0.0099
SNR	21.42	16.96	10.65	7.42	5.63

## Data Availability

The data that support the findings of this study are available upon request from the corresponding author.

## References

[1] Smith-Bindman R., Miglioretti D. L., Johnson E. (2012). Use of diagnostic imaging studies and associated radiation exposure for patients enrolled in large integrated health care systems. *JAMA*.

[2] Smith-Bindman R., Miglioretti D. L., Larson E. B. (2008). Rising use of diagnostic medical imaging in a large integrated health system. *Health Affairs*.

[3] Jones T., Townsend D. (2017). History and future technical innovation in positron emission tomography. *Journal of Medical Imaging*.

[4] Reinhard E., Heidrich W., Debevec P., Pattanaik S., Ward G., Myszkowski K. (2010). *High Dynamic Range Imaging: Acquisition, Display, and Image-Based Lighting*.

[5] Al-Qershi O. M., Khoo B. E. (2011). High capacity data hiding schemes for medical images based on difference expansion. *J SystSoftw*.

[6] Hashem I. A. T., Yaqoob I., Anuar N. B., Mokhtar S., Gani A., Ullah Khan S. (2015). The rise of “big data” on cloud computing: review and open research issues. *Information Systems*.

[7] House M. J., Bangma S. J., Thomas M. (2015). Texture-based classification of liver fibrosis using MRI. *Journal of Magnetic Resonance Imaging*.

[8] El Khaddar M. A., Harroud H., Boulmalf M., Elkoutbi M., Habbani A. Emerging wireless technologies in e-health trends, challenges, and framework design issues.

[9] Spaulding J., Noda H., Shirazi M. N., Kawaguchi E. (2002). BPCS steganography using EZW lossy compressed images. *Pattern Recognition Letters*.

[10] Mallat S. G. (2009). A theory for multiresolution signal decomposition: the wavelet representation. *IEEE Transactions on Pattern Analysis and Machine Intelligence*.

[11] Vetterli M., Herley C. (1992). Wavelets and filter banks: theory and design. *IEEE Transactions on Signal Processing*.

[12] Daubechies I. (1992). *Ten Lectures on Wavelets*.

[13] Juliet S., Rajsingh E. B., Ezra K. (2016). A novel medical image compression using Ripplet transform. *Journal of Real-Time Image Processing*.

[14] Cyriac M., Chellamuthu C. (2012). A novel visually lossless spatial domain approach for medical image compression. *European Journal of Scientific Research*.

[15] Brahimi T., Boubchir L., Fournier R., Naït-Ali A. (2017). An improved multimodal signal-image compression scheme with application to natural images and biomedical data. *Multimedia Tools and Applications*.

[16] Arif A. S., Mansor S., Logeswaran R., Karim H. A. (2015). Auto-shape lossless compression of pharynx and esophagus fluoroscopic images. *Journal of Medical Systems*.

[17] Das S., Kundu M. K. (2013). Effective management of medical information through ROI-lossless fragile image watermarking technique. *Computer Methods and Programs in Biomedicine*.

[18] Lucas L. F. R., Rodrigues N. M. M., da Silva Cruz L. A., de Faria S. M. M. (2017). Lossless compression of medical images using 3-d predictors. *IEEE Transactions on Medical Imaging*.

[19] Špelič D., Borut Ž (2012). Lossless compression of threshold-segmented medical images. *Journal of Medical Systems*.

[20] Anusuya V., Raghavan V. S., Kavitha G. (2014). Lossless compression on MRI images using SWT. *Journal of Digital Imaging*.

[21] Xiao B., Lu G., Zhang Y., Li W., Wang G. (2016). Lossless image compression based on integer Discrete Tchebichef Transform. *Neurocomputing*.

[22] Amri H., Khalfallah A., Gargouri M., Nebhani N., Lapayre J.-C., Bouhlel M.-S. (2017). Medical image compression approach based on image resizing, digital watermarking and lossless compression. *Journal of Signal Processing Systems*.

[23] Ramesh S. M., Shanmugam A. (2010). Medical image compression using wavelet decomposition for prediction method. *International Journal of Computer Science and Information Security*.

[24] Ibraheem M. S., Ahmed S. Z., Hachicha K., Hochberg S., Garda P. Medical images compression with clinical diagnostic quality using logarithmic DWT.

[25] Avramović A., Banjac G. (2012). On predictive-based lossless compression of images with higher bit depths. *Telfor Journal*.

[26] Bairagi V. K. (2015). Symmetry-based biomedical image compression. *Journal of Digital Imaging*.

[27] Zuo Z., Lan X., Deng L., Yao S., Wang X. (2015). An improved medical image compression technique with lossless region of interest. *Optik*.

[28] Srinivasan K., Dauwels J., RamasubbaReddy M. (2011). A two-dimensional approach for lossless EEG compression. *Biomedical Signal Processing and Control*.

[29] Taquet J., Labit C. (2012). Hierarchical oriented predictions for resolution scalable lossless and near-lossless compression of CT and MRI biomedical images. *IEEE Transactions on Image Processing*.

[30] Zanaty E. A., Ibrahim S. M. (2019). Medical image compression based on combining region growing and wavelet transform. *International Journal of Medical Imaging*.

[31] Roy V., Shukla S., Shukla P. K., Rawat P. (2017). Gaussian elimination-based novel canonical correlation analysis method for EEG motion artifact removal. *Journal of Healthcare Engineering*.

[32] Saxena A. K., Sinha S., Shukla P. (2018). Design and development of image security technique by using cryptography and steganography: a combine approach. *International Journal of Image, Graphics and Signal Processing*.

[33] Shukla P. K., Kaur Sandhu J., Ahirwar A., Ghai D., Maheshwary P., Shukla P. K. (2021). Multiobjective genetic algorithm and convolutional neural network based COVID-19 identification in chest X-ray images. *Mathematical Problems in Engineering*.

[34] Shukla P. K., Agrawal M., Khan A. U. (2019). Stock price prediction using technical indicators: a predictive model using optimal deep learning. *International Journal of Recent Technology and Engineering*.

[35] Tiwari P., Shukla P., Tuba M., Akashe S., Joshi A. (2020). Artificial neural network-based crop yield prediction using NDVI, SPI, VCI feature vectors. *Information and Communication Technology for Sustainable Development: Advances in Intelligent Systems and Computing*.

[36] Khambra G., Shukla P. (2021). Novel machine learning applications on fly ash based concrete: an overview. *Materials Today Proceedings*.

